The article "Identification of Food/Nonfood Visual Stimuli from Event-Related Brain Potentials" was published in 2021. Journal: Appl Bionics Biomech.

# Identification of Food/Nonfood Visual Stimuli from Event-Related Brain Potentials

**DOI:** 10.1155/2021/6472586

**Published:** 2021-09-23

**Authors:** Selen Güney, Sema Arslan, Adil Deniz Duru, Dilek Göksel Duru

**Affiliations:** ^1^Marmara University, Institute of Health Sciences, Istanbul, Turkey; ^2^Marmara University, Sports Science Faculty, Istanbul, Turkey; ^3^Department of Molecular Biotechnology, Turkish-German University, Istanbul, Turkey

## Abstract

Although food consumption is one of the most basic human behaviors, the factors underlying nutritional preferences are not yet clear. The use of classification algorithms can clarify the understanding of these factors. This study was aimed at measuring electrophysiological responses to food/nonfood stimuli and applying classification techniques to discriminate the responses using a single-sweep dataset. Twenty-one right-handed male athletes with body mass index (BMI) levels between 18.5% and 25% (mean age: 21.05 ± 2.5) participated in this study voluntarily. The participants were asked to focus on the food and nonfood images that were randomly presented on the monitor without performing any motor task, and EEG data have been collected using a 16-channel amplifier with a sampling rate of 1024 Hz. The SensoMotoric Instruments (SMI) iView XTM RED eye tracking technology was used simultaneously with the EEG to measure the participants' attention to the presented stimuli. Three datasets were generated using the amplitude, time-frequency decomposition, and time-frequency connectivity metrics of P300 and LPP components to separate food and nonfood stimuli. We have implemented *k*-nearest neighbor (kNN), support vector machine (SVM), Linear Discriminant Analysis (LDA), Logistic Regression (LR), Bayesian classifier, decision tree (DT), and Multilayer Perceptron (MLP) classifiers on these datasets. Finally, the response to food-related stimuli in the hunger state is discriminated from nonfood with an accuracy value close to 78% for each dataset. The results obtained in this study motivate us to employ classifier algorithms using the features obtained from single-trial measurements in amplitude and time-frequency space instead of applying more complex ones like connectivity metrics.

## 1. Introduction

Although food consumption is one of the most basic human behaviors, the factors underlying nutritional preferences are not yet apparent. Many factors, such as taste, texture, appearance, food deprivation, and smell of a meal, play an essential role in the attention to food [1–3]. Several studies point out increased attention given to food-related stimuli, mainly due to food deprivation [4, 5]. It is significant to identify both the activated brain regions and the temporal microstructure of the information flow between these regions to understand the neural foundations of a cognitive process such as the attention given to these types of stimuli [6]. Even though the methods of imaging (Magnetic Resonance Imaging (MRI), Functional Magnetic Resonance Imaging (fMRI), and Positron Emission Tomography (PET)) are very useful for showing changes in cerebral blood flow that occurred during cognitive processing, hemodynamic responses are insufficient to explain the temporal dynamics of fast electrophysiological activity in the neural network [6, 7]. Electroencephalogram (EEG) has a high temporal resolution that allows measurement of the brain's electrical activity [8–10] and varies concerning the presence of visual, somatosensory, and auditory stimuli [1, 11]. Event-Related Potential (ERP) recordings consist of sudden voltage fluctuations as a response to the stimulus [12, 13]. Researchers observed several ERP components according to the time delay after the occurrence of a stimulus. For instance, the P300 component, which is measured as a positive waveform approximately 300 ms after the stimulus, has been extensively studied in the literature due to its potential to reveal the dynamics of cognitive processes [14–19]. Moreover, Late Positive Potentials (LPP) are observed 550-700 ms after the stimulus that might be the projection of the focused attention or detailed stimulus analysis. Moreover, it reflects the conscious stimulus recognition phase. Wavelet transform (WT) is one of the methods that are capable of estimating the ERP components. WT has a more significant advantage than classical spectral analysis because it is suitable for the analysis of nonstationary signals in the time-frequency domain. WT can be used to analyze various transient events in biological signals with the structure of representation and feature extraction [20]. Each ERP component derived by WT can be associated with different situations and tasks [21–24]. In several studies, ERP components have been elucidated in response to food stimuli. For instance, Hachl et al. [25] conducted a study with a group of subjects who ate their last meal 3 hours or 6 hours before the ERP measurements where they used food images as stimuli. In another study, the effects of attention to food-related word stimuli in the absence of food were investigated [26]. Similarly, Channon and Hayward [27] investigated P300 and LPP responses to food and flower images in the hunger state. Furthermore, many researchers have conducted various Stroop studies in which the naming of the color of food words is used as stimuli [28–31]. Moreover, Kitamura et al. [32] observed the effect of hypoglycemic glucose drink intake on a P300 response. As a result, the P300 component varied as a response to food and nonfood stimuli in the hunger state. This variation motivated us to investigate the differences that occurred in the ERP components extracted from single-epoch electrical recordings.

In recent decades, the detection of the mental status via EEG measurements had been performed via the implementation of machine learning algorithms [33, 34]. In most of the studies, researchers computed the features from ongoing EEG time series, and those features were subjected to classifiers to detect whether the subject is normal or not [35, 36]. This procedure necessitated the use of known features while the modern approach, the deep learning mechanism, enables us to figure out the filters which can be used to classify the labelled measured data. A gross review has been given in [37] where the brain signals were used as inputs in various problems, including the seizure, emotion detection, motor imagery identification, and evoked potentials.

In addition, eye tracking technology is used in attention studies to understand whether the participant pays attention to the stimulus presented. Eye tracking technology is the name given to a set of methods and techniques used to detect and record the activity of eye movements [38]. Studies have shown that eye tracking data provide reliable measures of attention to the stimulus in complex situations [39, 40].

There are a few studies in the literature that classify food-related stimuli [32, 41]. Unfortunately, none of the previous studies have examined electrophysiological responses to food-related stimuli using classification techniques. This study is aimed at measuring electrophysiological responses to food/nonfood stimuli and applying classification techniques to discriminate the responses using a single-sweep time series.

## 2. Materials and Methods

### 2.1. Participants

Twenty-one right-handed male athletes with BMI levels between 18.5% and 25% (mean age: 21.05 ± 2.5) participated in this study voluntarily. All participants had a minimum training in a week of 10 hours and competed in karate or rowing. None of the participants had a lack of food intake, head injuries, neurological and psychiatric disorders, or other illness history.

### 2.2. Experimental Design

More specifically, participants were asked not to eat after 09.00 pm before the test day. We performed EEG measurements at 09.00-10.00 am before breakfast. Before the start of the experiment, we asked participants to focus on the food and nonfood images without large motor movements that can negatively affect the signal. We presented the stimuli randomly using in-house developed software. In our study, standardized and contrast-color-adjusted images were selected from the study of Charbonnier et al. to minimize the adverse effects of food images on the ERP [42]. In this study, we separated the images according to their nutrient content [43] into five groups. Since our aim is not to classify the response to the images through calorie content, we just separated the groups as food and nonfood ones. In the experiment, we have shown images for 800 ms and inserted a negligible time of two adjacent stimuli that are shown in Figure 1. The number of neutral images was 28 × 5, while it was 73 × 5 for food images. The resolution of the images was adjusted to 1280 × 1024.

### 2.3. Data Collection

We used a 16-channel V-AMP amplifier (Brain Products TM, Germany) with a sampling rate of 1024 Hz. In this study, we collected EEG from FP1, FP2, FP1, FP2, F3, Fz, F4, P3, P4, Pz, C3, C4, Cz, O1, O2 Oz, T7, and T8 channels with two electrodes as the reference and ground, as shown in Figure 2. Impedances of the channels have been kept below 5 khm.

The SensoMotoric Instruments (SMI) iView XTM RED eye tracking technology was used simultaneously with the EEG. A 22” LCD screen with 1920 × 1080 resolution and the eye-tracker system are shown in Figure 3. The frequency of the SMI eye-tracking system is 60 Hz, and it can record eye movements with a 0.5-degree recording error.

### 2.4. Data Analysis

Eye movements are analyzed to check if the subjects focused on the visual stimuli using SMI BeGaze (Behavioral and Gaze Analysis) software. Next, noisy components are removed from the EEG signal and the relevant properties of the data are extracted based on signal processing techniques. In this step, if the extracted features are not appropriate, inaccurate findings can be achieved. Thus, it is necessary to find and extract suitable features from the raw signals to obtain accurate classification results [44, 45]. The last step is the use of various machine learning techniques (like a decision tree and support vector machine) to classify the EEG signal using the characteristics obtained from the feature extraction process. Preprocessing of data is very substantial for improving the noise ratio of the EEG signal. We applied a low-pass filter at 40 Hz and a high-pass filter at 0.1 Hz. Artifacts have been marked on the EEG data and removed for further processing. After the preprocessing step, a total of 4754 single epochs remained. Next, EEG data are epoched with a length of 200 ms before and 800 ms post to each stimulus marker. In the second step, for both food images and nonfood images, the features are extracted using the data collected from 21 subjects. The feature vector consists of both time and frequency domain features. Datasets of essential features obtained from EEG for food and nonfood images are as follows: the amplitude, time-frequency power, and time-frequency connectivity metrics. Datasets have formed as follows. DataSet1: 16 attributes (16 electrodes) × 4754 row values are computed for the LPP and P300 amplitude. DataSet2: wavelet transform (WT) is used to compute 16 attributes (16 electrodes) × 4754 row values for each frequency band (delta, theta, alpha, beta, and gamma) for the LPP and P300. DataSet3: wavelet coherence is applied to form 120 attributes (15 × (15 + 1)/2 electrodes) × 4754 row values in each frequency band (delta, theta, alpha, beta, and gamma) for the LPP and P300.

The *k*-nearest neighbor (kNN), support vector machine (SVM), Linear Discriminant Analysis (LDA), Logistic Regression (LR), Bayesian classifier, decision tree (DT), and Multilayer Perceptron (MLP) classifiers are implemented using each dataset. The first classifier used in this study is the kNN, which is a nonparametric supervised learning algorithm. The new sample to be tested with the features extracted that occur during the classification is assigned to the most appropriate class according to its proximity to the *k*-nearest neighbors [46]. The second classifier, SVM, uses a distinctive hyperplane to determine classes. The hyperplane is the one that maximizes the margins using the distance from the nearest training points of the class. As a linear classifier, LDA (also known as Fisher's LDA) is an enhanced version of principal component analysis. The Bayesian classifier is a supervised statistical method for classification. It uses the probability to assign the most likely class of a given example described by its feature vector. MLP is a classifier based on artificial neural networks. The logistic regression used in this study is a statistical technique for binary classification. A tree-like structure containing the rules for classification in DT is produced using the mutual information hidden in the dataset. All of these classifiers were implemented in Python using the Scikit package.

## 3. Results

As a result of the analysis, the heat map of food/nonfood images obtained from the eye-tracking technology proves that the participants focused their attention on the presented images during the study as shown in Figures 4 and 5.

The grand average ERP components obtained from 21 subjects in the study are summarized in terms of P300 and LPP amplitudes as shown in Table 1. and Figure 6. We investigated the amplitude differences that occurred as a result of the presence of the food and nonfood stimuli using paired *t*-tests for each electrode.

Oz and T7 electrodes differed between food and nonfood stimuli significantly in the absence of a multiple test correction procedure while none of the electrodes' LPP components differed between stimuli. Further, this result motivated us to infer the mechanism of the measured ERP by the computation of the frequency decomposition. The increased occipital activity of the P300 observed concerning food stimuli agrees with our previous studies [47]. After the frequency decomposition of the EEG time series, we computed the statistical tests to elucidate the differences between food and nonfood stimuli. For the P300 component, in the delta band, Pz (*p* < 0.032) and Oz (*p* < 0.002); in the theta band, T7 (*p* < 0.03); and in the alpha band, FP2 (*p* < 0.014), electrodes differed between food and nonfood stimuli. On the other hand, for LPP, differences were observed just in the alpha band for Fp2 (*p* < 0.038), Fz (*p* < 0.016), T7 (*p* < 0.025), and T8 (*p* < 0.041).

Furthermore, we computed the coherence between the electrodes in each frequency band and performed *t*-tests to check the significance of the differences for food and nonfood stimuli. In the theta band, P300 coherence between Fp1 and Fp2 (*p* < 0.0003) and delta band LPP coherence of Fp2-Fz (*p* < 0.00037) are observed to differ between stimuli. After the descriptive investigation of the features, we focused on the classification procedures.

In this study, we achieved accuracy values close to 80% for the discrimination of the electrophysiological responses given to food-related stimuli versus nonfood stimuli in a hunger state, using various classification algorithms for datasets. The classification accuracy values are summarized in Tables 2–4 for the amplitudes of P300/LPP (DataSet1), for time-frequency-derived components of P300/LPP (DataSet2), and for connectivity metrics of the electrodes in the time-frequency domain of P300/LPP (DataSet3), respectively. A sample topography image is shown in Figure 7 for P300 and LPP while topographies regarding different time-frequency components are visualized in Figure 8.

We repeated the classification procedures based on individual subjects' data and reported the results (mean and standard deviation) in Table 5. In Figure 9, classification accuracy values of all algorithms are visualized.

## 4. Discussion

Up to our knowledge, the present study is the first one that classifies the electrophysiological responses to food and nonfood stimuli in a hunger state. For this, the first dataset consists of the amplitudes of the P300 and LPP components from single epochs. The dataset was formed by pooling the rows computed for each subject. As stated by Blankertz et al. [48], the investigation of ERP components from single-trial measurements is a complex problem because of trial variability and background noise. Thus, each row was normalized to avoid the amplitude differences within subjects and single-trial epochs. In the hunger state, P300 and LPP amplitudes were found to differ concerning food and nonfood stimuli in posterior regions [49]. Similar to this, Geisler and Polich reported P300 differences due to the food deprivation [31]. In contradiction to these findings, when the participants ingest hypoglycemic glucose, P300 changes were not observed [31]. In another study, LPP increased when the responses to food images and flower images were compared. In that study, P300 amplitude increased over the occipital, temporal, and centroparietal areas [26]. In our study, the maximum classification accuracy was 78% when the amplitudes of the P300 and LPP derived from single-trial measurements were used as features, separately. The differences in P300 or LPP components in the presence of the food/nonfood stimuli varied, as reported in previous studies. In ERP studies, averaging of the responses causes an increase in the signal-noise ratio of the signal and enhances the contrast between the cases.

However, in the concept of our study, a remarkable accuracy value (78%) has been obtained from the use of single-trial P300 and LPP amplitude components, separately. In the ERP literature, in a classification study, the average accuracy value increased to 86% based on the N170 component. In that study, single-trial measurements as responses to pictures having positive and negative emotions were the input data to the classifier [50]. Single-trial EEG measurements can provide valuable information in the presence of adequate contrast mechanisms. For instance, in the comparison of the resting-state EEG data with the brain dynamics measured during an increased mental workload state, high classification accuracy results are achieved [51]. In our study, the consistent accuracy values obtained using several techniques exhibit the limitation of the stimulus identification. DT outputs the lowest accuracy in classification, which might be due to the low number of levels of the tree.

For the ERP data collection, one needs to perform an averaging procedure over several responses given to the same or similar stimulus. Thus, conducting ERP experiments is a time-requiring process. On the other hand, in our study, we concentrated just on the single sweeps which last less than a second. So, the data that we need is limited by physiological mechanisms for the testing phase of the classification. Therefore, for real-time implementation, the minimum detection time can be thought of as the time needed to compute P300 and LPP features. On the other hand, the classification procedures consist of a training phase where several realizations of the labelled data are being used. For the estimation of the computational complexity, the number of features (*f*) and the number of samples (*n*) have a crucial role. For instance, in *k*-NN, in the test phase, the complexity is directly related to *f*∗*n*, while it is just affected by *f* in DT. Since the complexity values are on the order of the square of sample size, the training phase is time-consuming for DT, MLP, and SVM. On the other hand, LR is much faster. When we pool the data, our sample size becomes more than thousands.

## 5. Conclusion

In the ERP literature, the common sense is to analyze the electrical activity in different frequency bands. Thus, in the concept of this study, the time series were decomposed into a time-frequency space using wavelet transform. Moreover, the connectivity approach was adopted to multichannel ERP measurements in the time window of P300 and LPP to deduce the coherence information. Based on our findings, we can propose that the use of complex features is not necessary since the usage of them does not overcome the basic amplitude features.

There are still many gaps in our understanding of the brain responses given to visual stimuli. The concept of visual stimuli cannot directly be classified with high-accuracy values. On the other hand, it is more straightforward for mental illness detection or motor imagery studies. Thus, in future studies, one should focus on the feature engineering side of the EEG. In particular, deep learning with convolutional neural networks can be adopted to develop spatial filters on the topography images. This process may yield researchers to exhibit valuable information from the measured ERP signals.

## Figures and Tables

**Figure 1:** Graphical rendition of task.

**Figure 2:** 16 channel electrodes are distributed on the scalp.

**Figure 3:** SensoMotoric Instruments (SMI) Iview XTM RED and 22” LCD 1920 × 1080 screen.

**Figure 4:** Heat map of food images.

**Figure 5:** Heat map of nonfood images.

**Figure 6:** P300 and LPP amplitudes for food and nonfood stimuli.

**Figure 7:** Topographies of amplitude values of P300 and LPP.

**Figure 8:** Topographies of power values of P300 and LPP for each frequency band (*μ*V) (*δ* 0.5-4 Hz, *θ* 4-8 Hz, *α* 8-13 Hz, and *β* 13-30 Hz).

**Figure 9:** Classification accuracy for all algorithms with 10-fold cross-validation.

**Table 1:** Amplitudes of P300 and LPP components are summarized (microvolt).

Channel	P300 (Food) mean/std	P300 (Non-Food) mean/std	p	LPP (Food) mean/std	LPP (Non-Food) mean/std	p
Fp1	1.205/1.144	1.623/1.119	0.3695	2.315/1.142	2.114/1.091	0.7773
Fp2	-0.027 / 1.172	0.054/1.135	0.8795	1.020/1.171	0.445 /1.138	0.3008
F3	-6.537/1.155	-6.286/ 1.14	0.5663	-5.781/ 1.173	-5.822 /1.142	0.9162
Fz	7.298/ 1.008	7.462 / 1.001	0.7081	6.812 / 1.016	6.413 / 0.992	0.3246
F4	0.721/1.014	0.676 /1.019	0.9343	1.368 / 1.026	1.438/ 1.006	0.879
P3	4.107/ 1.008	4.461/ 0.989	0.3675	4.955 / 1.030	5.054/ 1.015	0.8533
P4	-15.839 / 1.282	-15.967/1.3	0.8282	-15.452/ 1.3	-14.816 / 1.329	0.2634
Pz	-8.574 / 1.186	-8.037/ 1.193	0.3823	-8.047/ 1.2	-8.468 / 1.197	0.4037
C3	2.556 / 0.960	3.079 / 0.954	0.2059	2.109 / 0.964	1.722 / 0.963	0.485
C4	-1.077 /0.946	-1.092/ 0.932	0.9672	-1.349 / 0.955	-1.37/0.938	0.9524
Cz	7.233 /0.963	7.405 /0.949	0.7175	6.215 / 0.964	6.177 / 0.940	0.9365
O1	1.193 / 0.999	0.899 / 0.996	0.3825	0.657 / 1.006	0.739 /1.035	0.8176
O2	4.099 / 0.982	3.856 / 0.989	0.5896	3.194 / 0.990	3.286 / 0.997	0.8204
Oz∗	5.218 / 0.952	4.275 /0.943	0.0122	4.752 /0.958	4.681 /0.953	0.8566
T7∗	-1.646 / 1.187	-2.662 / 1.151	0.0394	-2.08 / 1.19	-1.683 / 1.192	0.5251
T8	0.069/ 1.171	0.254 / 1.123	0.7408	-0.688 / 0.091	1.149 / 1.185	0.2419

**Table 2:** Accuracy of classifiers for P300 and LPP amplitude (%).

Method/Feature	P300	LPP
k-NN	76	76
LR	78	77
DT	65	66
LDA	78	77
NB	68	68
SVM	78	77
MLP	77	76

**Table 3:** Accuracy of classifiers for P300 and LPP power (%).

Method/Feature	P300 (%)	LPP (%)	P300 (%)	LPP (%)	P300 (%)	LPP(%)	P300 (%)	LPP (%)
k-NN	77	76	76	77	77	76	75	77
LR	77	76	76	77	78	76	76	78
DT	62	62	63	63	66	64	63	68
LDA	77	76	76	77	78	76	76	78
NB	74	73	76	76	78	76	76	78
SVM	77	76	76	77	78	76	76	78
MLP	77	75	76	77	78	76	76	77

**Table 4:** Accuracy of classifiers for P300 and LPP coherence (%).

Method/Feature	P300 (%)	LPP (%)	P300 (%)	LPP (%)	P300 (%)	LPP(%)	P300 (%)	LPP (%)
k-NN	77	76	76	77	77	77	77	77
LR	77	77	77	77	77	77	77	77
DT	64	62	63	64	63	64	64	65
LDA	77	77	77	77	77	77	77	77
NB	65	67	66	67	69	71	74	74
SVM	77	77	77	77	78	78	77	78
MLP	69	74	73	74	62	73	70	73

**Table 5:** The mean and standard deviation of accuracy values computed from each individual subject.

		Accuracy	k-NN	LR	DT	LDA	NB	SVM	MLP
Dataset 1	P300	Mean	73.7	75.1	71	75.1	71.7	73.9	61.6
		Std. Dev.	1.2	1.3	2.9	1.6	2.1	5.7	6.4
	LPP	Mean	74.1	75	70.6	75	71.8	76	61.5
		Std. Dev.	1.4	1.1	2.5	1.3	2	3.1	8.9

Dataset 2	P300 (Delta)	Mean	73.6	75.3	69.9	74.9	71.8	77.4	58.6
		Std. Dev.	1.6	1.6	2.9	1.5	2	0	13.5
	P300 (Theta)	Mean	73.6	74.9	70	74.9	71.3	77.4	54.1
		Std. Dev.	1.8	1.5	2.5	1.4	2.6	0	13.7
	P300 (Alpha)	Mean	73.5	74.8	70.7	74.9	70.9	77.4	59.2
		Std. Dev.	1.8	1.4	2.6	1.3	2.2	0	9.6
	P300 (Beta)	Mean	73.4	75	70.9	74.8	72.5	77.4	57.7
		Std. Dev.	1.7	1.7	2.6	1.5	2.3	0	9.6
	LPP (Delta)	Mean	73.7	65.2	69.2	59.3	62.1	70	58.1
		Std. Dev.	2.2	2.6	3.3	3.2	3.3	3	10.5
	LPP (Theta)	Mean	73.7	67.7	69.1	59.7	61.2	74.8	59.9
		Std. Dev.	1.5	2.5	3	3.4	5.1	1.5	9.7
	LPP (Alpha)	Mean	73.2	66.7	68.6	59.7	60.7	74	56.1
		Std. Dev.	2	2.7	2.7	2.8	5	2.2	8.9
	LPP (Beta)	Mean	73.6	67.3	67.6	59.8	61.8	75.6	61.7
		Std. Dev.	1.8	2.6	2.8	2.9	5.7	1.5	7.1

Dataset 3	P300 (Delta) Coh	Mean	73.3	65.7	69.8	58.4	60.8	69.3	55
		Std. Dev.	2	2.6	2.8	3.3	4.2	2.5	9.6
	P300 (Theta) Coh	Mean	73.6	67.6	68.5	58.1	61.8	74	58.1
		Std. Dev.	1.4	3.6	3.3	4.3	4.4	2.2	10.9
	P300 (Alpha) Coh	Mean	73.4	66.4	68.4	59.6	58.9	73.4	58.8
		Std. Dev.	1.7	3	2.3	3.3	5.9	1.7	7.4
	P300 (Beta) Coh	Mean	74.1	67.2	68.9	60.1	59.8	73.3	58.5
		Std. Dev.	2.1	2.4	2.5	3.9	5.4	2.3	9.6
	LPP (Delta) Coh	Mean	73.7	65.2	69.2	59.3	62.1	70	58.1
		Std. Dev.	2.2	2.6	3.3	3.2	3.3	3	10.5
	LPP (Theta) Coh	Mean	73.7	67.7	69.1	59.7	61.2	74.8	59.9
		Std. Dev.	1.5	2.5	3	3.4	5.1	1.5	9.7
	LPP (Alpha) Coh	Mean	73.2	66.7	68.6	59.7	60.7	74	56.1
		Std. Dev.	2	2.7	2.7	2.8	5	2.2	8.9
	LPP (Beta) Coh	Mean	73.6	67.3	67.6	59.8	61.8	75.6	61.7
		Std. Dev.	1.8	2.6	2.8	2.9	5.7	1.5	7.1

## Data Availability

The EEG and eye tracker data used to support the findings of this study are available from the corresponding author upon request.
